# Application of Biomaterials in Tendon Injury Healing and Adhesion in Sports

**DOI:** 10.1155/2022/5087468

**Published:** 2022-04-12

**Authors:** Rui Zhang

**Affiliations:** Bengbu Medical College Sports and Art Department, Bengbu 233000, Anhui, China

## Abstract

High-intensity sports make tendon injury of professional athletes occur frequently. However, tendon adhesion in the healing process of tendon injury seriously affects the normal functional training of athletes after rehabilitation. Therefore, based on the theory of tendon injury healing, the MRDM image data of tendon injury healing are obtained by using medical image analysis technology, and the useless image data are screened by using the RANSAC algorithm. Through the analysis of filtered MRDM image data, it is found that the application of biomaterials has a positive effect on promoting the stable healing of tendon. A multilevel model was used to evaluate the actual effect of several commonly used biomaterials in repairing tendon injury and adhesion. The results showed that sodium hyaluronate had the best repair effect on tendon injury.

## 1. Introduction

Sports are good for physical and mental health. After more than 100 years of development, there are many popular sports in the world, many of which have become one of the core events of the Olympic Games (Song) [1]. However, due to the high intensity of exercise itself, it is easy to cause damage to the body during exercise, among which tendon injury is the most prominent [2]. The following is tendon adhesion during tendon healing, which is a very common complication after tendon injury. Tendon adhesion directly affects the subsequent sports and technical competitions [3].

Therefore, how to prevent the healing of tendon injury has been a key research project of related researchers [4]. But so far, no simple and effective method for preventing tendon adhesion has been developed, and a stable healing of the tendon has been developed (Kang) [5]. With the development of modern medical technology, the use of biological materials to prevent the formation of tendon adhesion has made great progress (Zhang) [6].

After years of research, people have a clearer understanding of tendon adhesion (Gross and Hoffmann) [7]. First, the nutrient source required for tendon is that in addition to paratenon, retinaculum tendinum, and tendon bundle vessel, synovial is also a very important source of nutrients (Cheng and Jin) [8]. At the same time, tendon tissue itself can be self-healing. However, after the tendon injury, the tendon sheath is damaged and the synovial is reduced, resulting in insufficient nutrient supply, which slows the healing of the tendon tissue itself, and most of its repair process relies on peritendinous connective tissue for repair (Jia et al.) [9].

As a result, a large amount of scar tissue is produced, eventually forming adhesions (Yang et al.) [10]. Therefore, some scholars have proposed to intervene in the process of tendon healing through biological materials. The current mainstream practice is achieved through drug films (Nouiri et al.) [11]. The properties of this biomaterial are used to form a barrier to prevent the formation of adhesions, while at the same time directly affecting the healing of the tendons by drugs. In turn, a two-pronged approach is achieved to minimize the formation of adhesions (Han et al.) [12].

In this context, the application of biomaterials in the healing and adhesion of sports tendon injury was studied comprehensively. Through multiangle research and analysis, the advantages and disadvantages of current biomaterials for tendon adhesion repair are revealed, which provides the necessary theoretical basis for its future development (Zhang et al.) [13].

## 2. Related Work

For the repair principle of tendon, there are two different views in the academic world, one is the theory of endogenous healing and the other is the theory of exogenous healing (Lin et al.) [14]. Researchers supporting exogenous healing believe that tendons themselves are not self-healing and that fibroblasts that repair are produced from tendon sheaths and peritendon tissues (Moslehifard and Nokar) [15]. Adhesive bands from the tendon sheath and periorbital tissue are incorporated into the repair cells to achieve tendon repair (Koyanagi) [16]. Researchers believe that adhesions are necessary in the healing process, so it is impossible to completely prevent adhesions (Zhenyu et al.) [17]. Researchers who support the theory of endogenous healing have raised different opinions. During the study of the free tendon placed in the knee joint cavity, they found that the tendon survived on its own and also detected fibroblasts and newly formed collagen. These phenomena all indicate that tendons are self-healing (Guo et al.) [18]. In addition, researchers have found that human flexor tendons can be self-healing during the in vitro culture of human flexor tendons (Geng et al.) [19]. Researchers have also studied the collagen fibers secreted by tendon cells, which are found to be much larger than those produced by the outer membrane cells (Philip et al.) [20]. Moreover, when the newly formed collagen fibers are analyzed, it is found that the collagen fibers produced by the original tendon cells are arranged in the same manner. Therefore, some researchers believe that tendon cells themselves are also self-healing (as shown in Figure 1), can achieve self-proliferation, and self-repair by producing collagen by themselves.

According to research by relevant researchers, tendons can achieve endogenous healing. Therefore, improving the self-repairing efficiency of the tendon cells can effectively reduce the occurrence of adhesions. However, in the actual treatment process, endogenous healing and exogenous healing always exist simultaneously. This is because during the treatment of the tendon injury site, it is necessary to bring the drug into the tendon through the surrounding tissue. After the cut tendon sheath is sutured, there will still be some gaps. It may also be that after the synovial cells have fallen off, they are scattered in the synovial fluid and enter through them through the synovial. In another case, it is located in the tendon sheath. Due to the uneven cutting source and the internal friction of the sheath at the suture, it will cause a certain degree of wear on the inner surface of the sheath and then bring in foreign cells. Even if the tendon can be damaged and subcutaneous tissue, bone surface completely isolated, from the damaged place of the synovial sheath of the exogenous cells can still reach the damaged tendon, so there is no way to completely eliminate the entry of exogenous cells. As for the degree of exogenous healing is the majority or the degree of endogenous healing is the majority, it is judged based on the damage of the tendon, the nutritional status of the repair period, and the external environment. When the degree of exogenous healing is dominant, tendon adhesion will increase and vice versa. Taking into account the current level of medical technology, the best practice is to reduce exogenous healing as much as possible and increase the proportion of endogenous healing. Choosing the right biomaterial for treatment can achieve this goal well.

The properties of the biomaterial are utilized to form a barrier that prevents the formation of adhesions. At the same time, the drug directly affects the healing of the tendon, thereby achieving a two-pronged approach and minimizing the formation of adhesions. Since inflammation is highly likely to occur in areas where the tendon is damaged, inflammation causes the lymphatic vessels to be blocked by cellulose and proteins, resulting in hypoxia in the interior. Biomaterials allow the coverage area to maintain normal blood circulation and provide adequate oxygen supply for tendon repair. Not only that, but when inflammation occurs, it can destroy tissues such as giant cells, resulting in an increase in the concentration of the tissue fluid, an increase in the permeability of the capillaries, and an extravasation of a large amount of fluid, eventually resulting in edema. The use of biological materials here can accelerate blood circulation, resolve the problem of congestion, and eliminate edema. It is also possible to screen and isolate harmful active substances in blood vessels to ensure their recovery progress. In the process of using biological materials, due to its own physical characteristics, it can interfere with the transmission of painful impulses, thereby achieving the effect of relieving pain.

## 3. Theoretical Model Optimization

At present, the above tendon injury healing theory has been widely used in the medical field and has achieved good medical results. In order to verify the actual effect of biomaterials on the stable tendon healing of athletes, the MRDM image data of tendon injury healing were obtained by using medical image analysis technology to understand the tendon injury healing of patients (as shown in Figure 2). However, the collected data are mixed with a large number of worthless data. Therefore, it is necessary to use the RANSAC algorithm to filter worthless data.

The RANSAC algorithm is a data calculus method that uses an iterative random sampling method to extract and filter abnormal data to obtain a mathematical model. The implementation principle is mainly based on two different data types that exist in the sample data: (1) normal data model and (2) noise and abnormal data model. The algorithm believes that the data that cannot adapt to the mathematical model is mainly because the abnormal data may be caused by wrong assumptions in the process of mathematical model calculation or it is caused by the wrong way of calculation. However, these erroneous data often lack sufficient parameters to restore them. To this end, the algorithm restores its real data through multiple iterative screening methods. The RANSAC algorithm is mostly used in image processing in engineering. The basic implementation process is as follows:

It is needed to obtain necessary image data information, such as the edge of the object and the gray scale information. Whether the two information acquisitions are accurate or not will directly affect the accuracy of the detection. In general, when the system acquires graphics, it also needs to perform simple preliminary processing on the image, such as noise reduction. In this way, accurate information about the items to be inspected can be obtained accurately. The means of acquisition are mainly obtained by a CCD camera. Image enhancement is a very important step in image processing and one of the most used methods to improve image quality. There are two directions in this, one is to optimize the visual effect of the image and the other is to strengthen the characteristics of the image. Depending on the field of use, it can be divided into two types, one is airspace processing and the other is frequency domain processing. The former is processed directly on the image itself, while the latter is processed after the image is specially processed. The airspace processing formula is as follows:

(1) $$\begin{array}{c} g\left(x,y\right)=EH\left[f\left(x,y\right)\right], \end{array}$$

where the image before enhancement is *f*(*·*), *g*(*·*) is the enhanced image, and *EH* is the enhanced operation.

The edge information of the image is able to directly reflect the shape of the object, and its importance is obvious. Moreover, it can display most of the information of the item only by the partial image information. But its acquisition has a lot of difficulties. The data obtained by the edge in the system behave as a discontinuous gray value. This requires a special algorithm to calculate its edges. It is usually calculated using the first derivative and the second derivative. The gradient corresponds to the first derivative, and the gradient operator is the first derivative operator. For a continuous function *f*(*x*, *y*), its gradient at position (*x*, *y*) can be expressed as

(2) $$\begin{array}{c} \nabla f\left(x,y\right)=G\left(x,y\right)=\left[G_{x}\right.{\left.G_{y}\right]}^{T}=\left[\frac{\partial f}{\partial x}\right.{\left.\frac{\partial f}{\partial y}\right]}^{T}. \end{array}$$

A gradient is a vector whose amplitude and direction angle are

(3) $$\begin{array}{c} \left|\nabla f\right|=\left|G\left(x,y\right)\right|={\left[G_{x}^{2}+G_{y}^{2}\right]}^{\frac{1}{2}},\\ \phi \left(x,y\right)=\arctan\left(\frac{G_{y}}{G_{x}}\right). \end{array}$$

The approximate expression of the gradient is

(4) $$\begin{array}{c} G_{x}=f\left[i,j+1\right]-f\left[i,j\right],\\ G_{y}=f\left[i+1,j\right]-f\left[i,j\right]. \end{array}$$

Usually, in order to reduce the amount of calculation, the absolute value is usually used to approximate the gradient magnitude.

(5) $$\begin{array}{c} \left|G\left(x,y\right)\right|=\left|G_{x}\right|+\left|G_{y}\right|. \end{array}$$

When analyzing an image, the approximate value is usually calculated using a small area template tape measure. One template is used for each of A and B, which requires two templates. According to the size of different templates, the calculation properties are different. Therefore, there are Robert operators, Prewitt operators, and Sobel operators.

Roberts operator: the Robe operator approximates the magnitude of the continuous gradient of the edge point, and its convolution template is as follows:

(6) $$\begin{array}{c} G_{x}=\left[\begin{array}{cc} 1 & 0\\ 0 & -1 \end{array}\right],\\ G_{y}=\left[\begin{array}{cc} 0 & 1\\ -1 & 0 \end{array}\right]. \end{array}$$

The gradient templates in the horizontal and vertical directions of the Sobel operator are as follows:

(7) $$\begin{array}{c} G_{x}=\left[\begin{array}{ccc} -1 & 0 & 1\\ -2 & 0 & 2\\ -1 & 0 & 1 \end{array}\right],\\ G_{y}=\left[\begin{array}{ccc} 1 & 2 & 1\\ 0 & 0 & 0\\ -1 & -2 & -1 \end{array}\right]. \end{array}$$

The gradient template in the two directions of the Prewitt operator is as follows:

(8) $$\begin{array}{c} G_{x}=\left[\begin{array}{ccc} -1 & 0 & 1\\ -1 & 0 & 1\\ -1 & 0 & 1 \end{array}\right],\\ G_{y}=\left[\begin{array}{ccc} 1 & 1 & 1\\ 0 & 0 & 0\\ -1 & -1 & -1 \end{array}\right]. \end{array}$$

Then, the image content of the initial processing has been completed to extract corner points. It is assumed that variable *I*_*x*_ and variable *I*_y_ are used to represent the first-order partial derivative of image *I* in two different aspects of Cartesian coordinate *x* and y axes. Then, the function *w*(*x*, *y*) can be used to represent a two-dimensional Gaussian smoothing function on Cartesian coordinates. The calculation process of this function is shown in the following two formulas:

(9) $$\begin{array}{c} M=\sum_{x,y}w\left(x,y\right)\left[\begin{array}{cc} \overset{2}{\underset{x}{I}} & I_{x}I_{y}\\ I_{x}I_{y} & \overset{2}{\underset{y}{I}} \end{array}\right],\\ R=\det M-k\cdot {\left(\text{trace}M\right)}^{2},k=0.04∼0.2. \end{array}$$

Solving formula (15) can yield a specific number for each corner *R* on the image. Then, using the normalization idea to match the calculated corner points, the image corner point value can be obtained. The matching calculation equation is as follows:

(10) $$\begin{array}{c} NCC=\frac{\sum_{i}\left(I_{1}\left(x_{i},y_{i}\right)-u_{1}\right)\left(I_{2}\left(x_{i},y_{i}\right)-u_{2}\right)}{\sqrt{\sum_{i}{\left(I_{1}\left(x_{i},y_{i}\right)-u_{1}\right)}^{2}\sum_{i}{\left(I_{2}\left(x_{i},y_{i}\right)-u_{2}\right)}^{2}}}. \end{array}$$

It is worth noting that the results obtained by using the normalized thought tend to be mixed with some singularities. These singularities are the anomalous data belonging to the corner values of the image that are noisy and cannot be normally described by the mathematical model. Therefore, it is necessary to use the RANSAC algorithm to purify the image corner values (as shown in Figure 3). In the process of purification, the images should be considered separately according to the three color channels of red, green, and blue. Then, there is the following linear algebraic equation:

(11) $$\begin{array}{c} \left(\begin{array}{c} R_{2}\\ G_{2}\\ B_{2} \end{array}\right)=\left(\begin{array}{ccc} c_{r} & 0 & 0\\ 0 & c_{g} & 0\\ 0 & 0 & c_{b} \end{array}\right)\cdot \left(\begin{array}{c} R_{1}\\ G_{1}\\ B_{1} \end{array}\right)+\left(\begin{array}{c} d_{r}\\ d_{g}\\ d{}_{b} \end{array}\right). \end{array}$$

In the above formula, the variable *R*_2_, the variable *G*_2_, and the variable *B*_2_, respectively, represent three color channels of red, green, and blue of the image. The variable (*R*_2_, *R*_1_)_n_ is mainly used to represent the transformation parameters of the linear equation (c, d). At this point, the purification is done by iterative summation as follows:

(12) $$\begin{array}{c} E=\sum T\left(d_{n}{}^{2}\right), \end{array}$$

In the above formula, when the condition satisfies *d*_*n*_^2^ < Thre^2^, then *T*(*d*_*n*_^2^)=*d*_*n*_^2^, otherwise *T*(*d*_*n*_^2^)=Thre^2^. Filter the corner points of the image that meet the conditions and continue the iterative calculation. The entire purification process is completed until the value of E does not change significantly. At this point, all data points belong to the data that can be normally described by the mathematical model. Finally, it is necessary to split the image. The effect of image segmentation is good or not will directly determine whether the analysis of the image is in place or not.

The similarity calculation is performed after the image is segmented, and the predetermined image in the database and the matching are performed according to the calculated result. The matching result of the image is extremely characteristic. The following function is used to measure the similarity between *T* and *f*:

(13) $$\begin{array}{c} SE\left(x,y\right)=\sum_{i=1}^{N}\sum_{j=1}^{N}{\left[f\left(x-i,y-j\right)-T\left(i,j\right)\right]}^{2}, \end{array}$$

where the size of the image is *N* × *N*, the above formula provides a measure of the degree of matching between the image *T* and the subgraph *f* at the (*x*, *y*) coordinate. Expand the above formula to calculate the matching result:

(14) $$\begin{array}{c} SE\left(x,y\right)=\sum_{i=1}^{N}\sum_{j=1}^{N}f^{2}\left(x-i,y-j\right)-2\sum_{i=1}^{N}\sum_{j=1}^{N}f\left(x-i,y-j\right)T\left(i,j\right)+\sum_{i=1}^{N}\sum_{j=1}^{N}T^{2}\left(i,j\right). \end{array}$$

## 4. Experimental Results and Analysis

Sports posture is complex, and the amount of exercise is large. Because of the above reasons, professional athletes often have tendon injury in the process of sports. Tendon adhesion is a very common complication after tendon injury in the process of tendon healing and temporarily unable to recover, will affect the athlete's competition and training in varying degrees. Based on the above reasons and based on the theory of tendon injury healing, the MRDM image data of tendon injury healing were obtained by using medical image analysis technology, and the worthless image data were screened by using the RANSAC algorithm. Then, through the analysis of the filtered MRDM image data, it is found that the application of biomaterials can actively promote the stable healing of tendon. Finally, the clinical application of biomaterials is listed, and the actual effect of several commonly used biomaterials to repair tendon injury and adhesion is evaluated by using the multilevel comprehensive evaluation model.

At present, the biological materials commonly used in medical clinics for repairing tendon injury healing adhesions (as shown in Figure 4) are mainly the following: (1) Chitosan: the biomaterial can effectively inactivate the fibroblasts at the site of the damage of the organism and inhibit the growth cycle of the fibroblasts. Furthermore, the proliferation time of endothelial cells is reserved for growth and self-repair of the human body. (2) Absorbable antiadhesion film: the biomaterial can also inactivate fibroblasts at the site of damage to the organism, and it can also act as a barrier to aid in the repair of the tendon. In addition, the absorbable antiadhesion film belongs to a biological material that can be absorbed and degraded by the living body. (3) Sodium hyaluronate: the biomaterial is a liquid material composed of a sodium salt and has high biocompatibility.

In order to more accurately screen out the biomaterials with the best effect on repairing tendon injury, the multilevel fuzzy comprehensive evaluation model is used to evaluate the actual effects of the above three biomaterials for repairing tendon injury healing. The multilevel fuzzy comprehensive evaluation model is an evaluation method based on cognitive science and fuzzy mathematics. The specific form is as follows:

(15) $$\begin{array}{c} \left(\begin{array}{cccc} a_{1,1} & a_{1,2} & \ldots & a_{1,n}\\ a_{2,1} & a_{2,2} & \ldots & a_{2,n}\\ \cdot & \cdot & \cdot & \cdot \\ a_{n,1} & a_{n,1} & \ldots & a_{n,n} \end{array}\right). \end{array}$$

In the formula, *ai*, *j* represents the relative weight of indicator *ai* relative to indicator *aj*.

Calculate the product of each row element of the judgment matrix R,

(16) $$\begin{array}{c} M_{i}=\prod_{j=1}^{n}B_{ij},i=1,2,\ldots ,n. \end{array}$$

Calculate the root in the times *n* of *M*_*i*_,

(17) $$\begin{array}{c} \bar{w_{i}}={\left(M_{i}\right)}^{\frac{1}{n}},i=1,2,\ldots ,n. \end{array}$$

The normalization of $\bar{w_{i}}$ is as follows:

(18) $$\begin{array}{c} w_{i}-\frac{\bar{w_{i}}}{\sum_{i=1}^{n}\bar{w_{i}}},i=1,2,\ldots ,n. \end{array}$$

Then, the weighting vector is *w*=[*w*_1_, *w*_2_,…,*w*_4_]^*T*^.

The target criterion layer weight vector obtained according to the above method is as follows:

(19) $$\begin{array}{c} W=\left(w_{1},w_{2},w_{3},\ldots ,w_{k}\right). \end{array}$$

*w*_*i*_ is the relative weight of the criterion layer indicator i in the criterion layer.

For the criterion level indicator of number k, the weight of the measure level under each criterion is as follows:

(20) $$\begin{array}{c} W_{k}=\left(w_{k1},w_{k2},w_{k3},\ldots ,w_{kp}\right). \end{array}$$

In the hierarchical structure, the comprehensive weight calculation operator of the measure indicator j under criterion i is as follows:

(21) $$\begin{array}{c} w_{i,j}=w_{i}\cdot w_{j}. \end{array}$$

After obtaining the weights of the respective indicators, the evaluation score can be finally calculated by multiplying the evaluation values. The calculation operator is as follows:

(22) $$\begin{array}{c} Ea=\left(w_{p,1},w_{p,2},\ldots ,w_{p,n}\right){\left(v_{p,1},v_{p,2},\ldots v_{p,n}\right)}^{T}. \end{array}$$

*w*_*p*,*i*_ is the comprehensive weight of the lowest level indicator i, and *w*_*p*,*i*_ is its evaluation score.

Substituting the data information recorded during the experiment into the above equation can obtain the evaluation result as shown in Figure 5. The data in the figure indicate that the three kinds of sodium hyaluronate in the biomaterials for repairing tendon injury healing have the best tendon damage repair effect.

In order to observe the effect of hyaluronic acid with different molecular weight, Hyalgan and Synvisc were used to evaluate the efficacy of knee osteoarthritis [21]. The rabbit knee osteoarthritis model was made by unilateral anterior cruciate ligament transection. Two weeks after operation, it was randomly divided into group A, group B, and control group (group C). Group A was given Hyalgan 0 2 ml, group B was given Synvisc 0 2 ml, and group C was given 0.2 ml of 0.9% sodium chloride injection. All patients received intra-articular injection once a week for 4 weeks. Three groups of animals were killed 10 weeks after operation, and articular cartilage was taken for gross observation and histological observation under the microscope. Mankin score—the results showed that group A and group B were significantly lighter than group C (*P* < 0.05), while group B was significantly lighter than group A (*P* < 0.05). Synvisc, a hyaluronic acid preparation with high molecular weight, has better short-term therapeutic effect on rabbit knee osteoarthritis than Hyalgan [22].

## 5. Conclusion

Professional athletes often encounter tendon injury in the process of exercise and then tendon adhesion occurs in the process of tendon healing. Tendon injury is a common complication after tendon injury. It is difficult to recover after a period of time, which has different effects on athletes' competition and training. Based on the above reasons, the theory of tendon injury healing has been deeply studied, and it is found that the biological barrier of biomaterials can effectively promote tendon repair and self-healing. In order to verify the actual effect of biomaterials on tendon healing, MRDM image data of tendon injury healing were obtained by medical image analysis technology for research and observation. The acquired MRDM image data contain a lot of useless information. For this reason, the RANSAC algorithm is used to filter the worthless image data and then in-depth analysis is carried out. The application of biomaterials can actively promote the stable healing of tendon. Then, the multilevel model was used to evaluate the actual effect of several biomaterials: (1) chitosan; (2) absorbable antiadhesion membrane; and (3) sodium hyaluronate, which is commonly used in the clinic to repair tendon injury and heal adhesion. The results showed that sodium hyaluronate was the best of the three biomaterials for tendon healing.

## Figures and Tables

**Figure 1:** Self-repair of collagen fibers produced by tendon cells.

**Figure 2:** The healing of tendon injury was obtained by medical image analysis.

**Figure 3:** In the process of purification, the image should be considered separately according to the red, green, and blue channels.

**Figure 4:** It is a common biological material used in repairing tendon injury and adhesion.

**Figure 5:** Evaluation of growth status of agrobacterium bisporus.

## Data Availability

The data used in this paper to support the results of this study are included in this paper.
